# Rutin: A Flavonoid as an Effective Sensitizer for Anticancer Therapy; Insights into Multifaceted Mechanisms and Applicability for Combination Therapy

**DOI:** 10.1155/2021/9913179

**Published:** 2021-08-23

**Authors:** Atefeh Satari, Sorayya Ghasemi, Solomon Habtemariam, Shirin Asgharian, Zahra Lorigooini

**Affiliations:** ^1^Cellular and Molecular Research Center, Basic Health Sciences Institute, Shahrekord University of Medical Sciences, Shahrekord, Iran; ^2^Pharmacognosy Research Laboratories and Herbal Analysis Services, University of Greenwich, Central Avenue, Chatham-Maritime, Kent ME4 4TB, UK; ^3^Medical Plants Research Center, Basic Health Sciences Institute, Shahrekord University of Medical Sciences, Shahrekord, Iran

## Abstract

Rutin is a unique antioxidant flavonoid that is mainly found in fruit, vegetables, cereals, and many other plant-based human diets. This review aims to highlight the *in vitro* anticancer properties of rutin including combination therapeutic strategies. Literature resources were gathered through PubMed, Scopus, Web of Science, and Google Scholar databases that cover the period of 1995–2021. Rutin is demonstrated to inhibit the proliferation of breast, colon, lung, and prostate cancers and other tumors. Furthermore, rutin alone or in combination with other therapeutic agents has been shown to regulate several signalling pathways involving the Ras/Raf and PI3K/Akt, MAPK, and TGF-*β*2/Smad2/3Akt/PTEN, etc., which are related to the processes of carcinogenesis and induction of apoptosis. The combination of rutin with other chemotherapy drugs may benefit on prevention of tumor cells by decreasing drug resistance and chemotherapy side effects. Moreover, rutin induces apoptosis synergistically with the therapeutic agent. More *in vivo* and clinical data are however needed to evaluate the true potential of rutin as an anticancer agent as an adjuvant. The present review highlights the effects of rutin which can be a promising candidate in combination with other antitumor drugs or alone for cancer treatment *in vitro*. Also, rutin can lead to decrease in drug resistance and chemotherapeutic side effects.

## 1. Introduction

### 1.1. Chemical Structure of Rutin as a Flavonoid

The 15-carbon basic structure of flavonoids consists of a three-ring system arranged as C6-C3-C6. This normally includes two aromatic rings (rings A and B) often in polyphenolic forms joined together with a three-carbon chain to form the third ring (ring C) in many flavonoids. Depending on the oxidation state, presence or absence of double bond, and the way ring C is connected with ring B, flavonoids are classified into different families such as flavonols, flavones, and flavanones [1]. Biosynthetically, the first group of flavonoids that are considered precursors are the chalcones. Naringenin chalcone is one of the first chalcone derivatives to be produced naturally and could give rise to flavanones such as naringenin (Figure 1). Flavones such as apigenin have low toxicity and multiple beneficial bioactivities. Rutin possess a double bond in ring C and further hydroxylation at the C-3 position gives rise to flavonols such as rutin and kaempferol (Figure 1). Quercetin is a derivative of flavonols with diorthohydroxyl group in the ring, while its ruinoside derivative at the C-3 position is called rutin (Figure 1) [2].

Glycosyl flavonoids include the C-glycosides and O-glycosides depending on the sugar attachment bound as a C–C bond or C–O bond. Several C-glycoside flavones (e.g., at C-6 or C-8 position) such as rutin are more impressive in biological activities than O-glycosides flavone isomers [3, 4]. The various biological activities of flavonoids include therapeutic implications against diseases such as cancer, depression, diabetes, dementia, lupus, autism, and heart disease. They also exhibit strong antioxidative activity which is often considered as a mechanism of action for their healing functions in irregular biological systems such as cancer cells. Flavonoids such as rutin are found mainly in fruits, vegetables, grains, and many other human diets [5–7]. Several studies have shown that flavonoids as polyphenolic compounds possess antiproliferative and cytoprotective effects in addition to induction of apoptosis in different cancer cell lines [8].

Some flavonoids have been shown to regulate several signal proto-oncogene pathways. Proto-oncogenes have been shown to encode cell surface receptors, nuclear proteins, membrane proteins, growth factors, and phosphokinases. C-Fos, c-Jun, and c-Myc as three important proto-oncogenes are associated with both processes of carcinogenesis and inflammation. In the same way, rutin induced cytotoxicity through genotoxicity, mitochondrial apoptotic pathway, and relatively upstream apoptotic factors, including reduction of ROS generation and induction of antioxidant enzyme (AOE) (Figure 2) [9, 10].

Among the nuclear proteins coded by proto-oncogenes (c-Onc) are c-Myc, c-Fos, and c-Jun. These proteins have the potential to regulate other genes directly or indirectly, thereby influencing some gene expressions and apoptosis. This review aims to highlight the *in vitro* anticancer properties of rutin including combination therapeutic strategies: A Novel Treatment Strategy for Cancer Treatment.

### 1.2. Natural Occurrence and General Pharmacological Effects of Rutin

The metabolism, absorption, and antioxidant activity of flavonoids significantly differ from each other based on structural variations including the presence, nature, and position of glycosylation [11]. Among the phytochemicals with anticancer effects, rutin (3,3′,4′,5,7-pentahydroxyflavone-3-rhamnoglucoside: Figure 3) is one of the highly potent antioxidant agents, with some other biochemical activities in cancer prevention and treatment. Due to these biological effects, rutin is also known as vitamin P [5, 12]. More than 130 therapeutic drugs that have been existed are containing rutin in their structure. It is found in plants such as buckwheat, green tea, and apples and is widely used as medicine in China. Buckwheat is one of the major sources of rutin [13, 14]. The origin of rutin from the buckwheat plant can go back to the 1940s when buckwheat was used for medicinal purposes in the United States. Notably, the leaves and flowers of the plant were found to be in the highest concentration, nearly 2–10% of plant weight. The content of rutin at various parts of the plant considerably depends on its geographical source and genetic type [15, 16]. Moreover, it is demonstrated that more than 70 plant species are good sources of rutin and these include *Ruta graveolens* L. (Rutaceae) and *Sophora japonica* L. (Fabaceae), *Strelitzia reginae* Banks ex Aiton (Strelitziaceae), *Maranta leuconeura* (Marantaceae), *Orchidantha maxillarioides* (Lowiaceae), *Eucalyptus* spp. (Myrtaceae), *Canna indica* L. (Cannaceae), and *Canna edulis* Ker Gawl. (Cannaceae) [15, 17]. Up to 1.5% of rutin could also be extracted from tobacco leaves [18]. The biosynthesis of rutin is regulated by ultraviolet light and its accumulation serves as a protection. In this connection, when dill cell cultures were subjected to sunlight, the prominent flavonoid synthesized was shown to be quercetin-3-O-*β*-glucuronide. Both rutin and quercetin are major sources of pharmaceutical products for phytotherapy [19, 20].

Many studies revealed rutin possesses anti-inflammatory, anticarcinogenic, neuroprotection, antiproliferative, antimetastatic, and antioxidative stress effects via inhibiting lipid peroxidation and amelioration of oxidative stress [21, 22]. Reactive oxygen species (ROS) can damage DNA, chromosomal mutations, unregulated gene expressions, cell division, and cell growth. Also, they could reduce the activities of some proteins involved in the antioxidant systems [23, 24]. Several studies have reported that ROS are associated with some tumors such as colon cancer, hepatocellular carcinoma, leukaemia, neuroblastoma, lung cancer, and breast cancer [12, 25–27]. Lipid peroxidation is the process by which oxygen combines with lipids to produce lipid hydroperoxides through the intermediate formation of peroxyl radicals and the cleavage of hydrogen. Unless checked by antioxidants such as rutin, lipid peroxidation can play a significant pathological role. Previous studies have shown that modified lipid composition could lead to cell apoptosis and other effects that could be targeted by rutin. Furthermore, rutin eliminating edema and reduction in sensitivity reduced ischemia-reperfusion damage. Rutin provides pharmacological information via platelet aggregation and cyclooxygenase-1 inhibition and its downstream pathway (Figure 4) [28, 29].

Therefore, rutin is considered a promising natural product in cancer prevention not only for its known efficacy but also accessibility and limited side effects.

## 2. Anticancer Properties of Rutin through Modulation of Signalling Pathways

Cancer is associated with the free radical generation and oxidative stress, fatty acid synthase (FAS) gene expression, and other mechanisms that lead to tumor via multiple modifications and mutations in cell proliferation and apoptosis genes controlling [1, 5]. Among the flavonoids with anticancer effects, rutin has one of the most widespread uses as an antioxidant and as an antitumor agent among the flavonoids because of its abundance in the human diet such as fruits and vegetables [30]. Here is a summary of its most important anticancer functions.

In some types of cancer, an oncogenic change induces an inflammatory microenvironment that promotes the development of cancers. The molecular pathways of this cancer-related inflammation are now being unravelled, resulting in the identification of new target molecules that could lead to improved diagnosis and treatment. There is also evidences to suggest that rutin exerts anti-inflammatory effects by downregulating the expression of cyclooxygenase-2, inducible nitric oxide synthase (iNOS), and suppression of lipid peroxidation. Also, rutin suppresses proinflammatory cytokines secretion [5, 31]. Nitric oxide is synthesized by a family of isoenzymes in normal cells. The high expression of stimulation nitric oxide synthase (NOS) via myeloid-derived suppressor cells (MDSCs) is a major signal of defence mechanism in cancer. NOS is also expressed by *γδ* T cells by contributing to their polarization to a protumor phenotype in cancer. Moreover, it has been indicated that rutin modulates activators of transcription, mitogen‐activated protein kinase (MAPK), PI3K/Akt, and Wnt/*β*‐catenin signalling cascades and Janus kinase/signal transducers in carcinogenic cells. The Ras/Raf and PI3K/Akt, MAPK, and TGF-*β*2/Smad2/3Akt/PTEN signalling pathways are stimulated through the epidermal growth factor (EGF) signalling pathway [14, 32, 33]. Rutin has been demonstrated to directly bind to the EGF receptor (EGFR) protein and arrest the downstream signalling factors [5]. They demonstrated that rutin reduces the expression of miR‐22‐5p an important microRNA in increasing the levels of RAP1/ERK signalling pathway‐related proteins that lead to apoptosis in *in vitro* and *in vivo* studies via *Rap1a. Rap1a* is one of the target genes of miR‐22‐5p [14, 34]. The present review highlights the anticancer potentials of rutin on cancer cell lines such as the colon, lung, breast, prostate, and HepG2 through various known molecular mechanisms including modulation of apoptosis genes in *in vitro* experimental models (Tables 1 and 2) [57].

### 2.1. Rutin Induces Apoptosis and Arrests the Cell Cycle in Tumor Cells

Apoptosis is a process of eliminating damaged cells and is executed by a family of caspases. It is regulated by apoptotic gene expression such as *p*53 and Bax [58]. The *p*53 gene mutation is the most common genetic irregularities related to apoptosis in human tumors. Rutin (900 *μ*m) was found to downregulate the expression of mutant *p*53 protein in human prostate cancer cell lines (DU-145, PC-3, and LNCaP) [21, 59].

The G1 and G2 phases of the cell cycle controlled by the *p*53 gene are a main regulatory mechanism in cellular proliferation [20]. Many studies demonstrated that rutin increases glutathione S-transferase P1 (GSTP1) polymorphism, Cyp1A1 cytochrome P450 (CYP1A1, CYP2D6) polymorphisms (inhibitory effect of antitumor genes), *p*53 (apoptosis gene expression), and Nqo-1 (antioxidant enzyme) leading to cell cycle arrest and consequently induction of apoptosis [21, 46, 60]. Also, it was reported that rutin could decrease Bcl-2 antiapoptosis gene expression and Bcl-2/Bax ratio along with a reduction in the levels of MYCN mRNA [61] (Figure 5). Moreover, other studies suggest that rutin can inhibit and regulate the cell cycle in the G2 and G1 phases. It stimulates apoptosis and decreases some of the oncogenic pathways including NF-*κβ* pathway and phosphorylation of the *p*38 MAP kinase [60, 62]. Therefore, these studies brought to light the unique roles of rutin in the prevention and treatment of cancer via the control of cellular proliferation and apoptosis induction [9].

### 2.2. Anticancer Effect of Rutin: Single Therapy on Cancer Cell Lines

There are numerous *in vitro* studies that investigate the effect of rutin on the proliferation of cancer cell lines, such as the breast, colon, prostate, and lung. Rutin caused growth inhibition in human glioblastoma cell lines through induction of apoptosis and G2/M phase cell cycle arrest, as well as regulation of expression of the pro- and antiapoptotic genes (Bcl-2, Cas-3, Bax, and TP53). It also reduced mitochondrial membrane potential [62]. Rutin (400–700 mM/ml) has shown *in vitro* antiangiogenic properties on SW480 (human colon adenocarcinoma cell line) through cell cycle arrest at G1 phase and regulation of microRNAs (miRNAs), long noncoding RNAs (lncRNAs), messenger RNAs (mRNAs), and transcription factors (TFs) [26, 31]. Rutin as well as other antioxidants such as gallic acid, chlorogenic acid, coumaric acid, quercetin, and ferulic acid also induced cell apoptosis via a caspase-independent pathway [63]. In another cancer, osteosarcoma, it was further reported that rutin can stimulate osteoblast in human MG-63 cells [31, 64]. Other studies demonstrate that rutin exerts a notable reduction in tumor extent on human leukaemia (HL-60) and hepatic cells [65–67]. Also, rutin significantly inhibited the growth of LAN-5 and neuroblastoma cells through induction of apoptosis and cycle arrest at the G2/M phase [61]. Some studies indicated that rutin (810 *μ*m) can cause a decrease in viability and consequently induce apoptosis in human liver cells [66, 68]. In breast cancer MDA-MB-231 cells, MCF‐7 cell line, and HTC hepatic cells, rutin has been shown to modulate the Wnt, JAK-STAT, EGF signalling, AP-1, NF-*κ*B, and Akt [69, 70]. Therapeutically controlling cell signalling using different antioxidants has been demonstrated to have promise in cancer though it still needs more research [69]. In studies conducted by Karakurt on human hepatocytes (HepG2), rutin showed a regulatory role in the expression of cytochrome P450 and antioxidant enzymes [60]. Another study indicated a defensive effect of rutin on LLC‐PK1 cells (a porcine renal tubular epithelial cell line) that caused cell death and production of intracellular ROS [5, 71]. It also exerts *in vitro* cytotoxic effects on prostate cancer cells via increased caspase activity and apoptosis [72]. Moreover, rutin could be a candidate therapeutic agent for the treatment of human lung (A549) and colon (HT-29 and Caco-2) cancer cell lines by decreasing cell viability [53, 73]. Rutin treatment could significantly inhibit endothelial cell proliferation *in vitro* with the implication of angiogenesis inhibition [56]. So, rutin seems to be useful as an adjuvant in cancer therapy and the evidence shows that it alone has some anticancer potentials.

### 2.3. Rutin as a Combination Therapy with Antioxidants or Herbal Ingredients in Cancer Cells *In Vitro*

Combination therapy, the main treatment strategy that combines two or more therapeutic agents, is recently used by many investigators for cancer therapy. It has been shown that the mixture of antioxidants can promote antiproliferative, anticarcinogenic effects when compared to the monotherapy approach in cancer [48, 74, 75] (Table 1). The results have shown that rutin prenanoemulsion could inhibit cancer cells such as lung cancer cell line (A549) and colon cancer cell line. Also, the effects of rutin with antioxidants prevented protein modifications by lipid peroxidation products. Further, it induced rutin-protein adduct formation, which supports intra/extracellular signalling and the Nrf2/ARE antioxidant pathway, contributing to the protective effects against UV-induced oxidative stress [76].

Regulation of cellular signalling pathways such as Wnt/*β*‐catenin, *p*53‐independent pathway, apoptosis, JAK/STAT, PI3K/Akt, and MAPK as well as NF‐*κ*B signalling pathways helps to mediate the anticancer effects of rutin. Exploration of these antitumor mechanisms can facilitate the development of this beneficial compound for its application in the treatment of cancers [77–79].

### 2.4. Rutin in Combination with Chemotherapy Drugs: *In Vitro* Studies

Randomized clinical trials have shown that the administration of antioxidants with chemotherapeutic drugs offers the possibility of better tumor protection and survival [74, 80]. Also, previous studies have demonstrated that rutin in combination with drugs can reduce the proliferation of many cancer cells through activation of apoptosis and arrest the cell cycle and many other mechanisms (Table 2). Therefore, the present review aimed to show the synergistic effects of rutin with anticancer drugs in cancer cell lines (Table 2). Rutin was demonstrated to target various inflammatory, apoptotic, autophagic, and angiogenic signalling mediators, including nuclear factor-*κ*B, tumor necrosis factor-*α*, interleukins, light chain 3/Beclin, B cell lymphoma 2 (Bcl-2), Bcl-2 associated X protein, caspases, and vascular endothelial growth factor [40, 81]. A critical analysis of the anticancer potential of rutin and associated molecular targets among various cancer types has not been performed previously. Moreover, combination therapy can lead to a decrease in drug resistance and chemotherapeutic side effects [40, 78–82].

## 3. Applications of Novel Drugs and Limitations Associated with the Use of Some Flavonoids Such as Rutin

Great advances have been made on the development of novel drug combination systems for plant actives. The variety of novel herbal formulations like Rutin as a promising candidate in combination with other antitumor drugs or alone has been reported for cancer treatment by decreasing the exposure in normal tissues exploiting enhanced permeability and retention effect phenomenon by utilizing targeting strategies. Also, improve the efficacy of herbal cosmetic formulations on the human body. The mentioned formulations demonstrated that they have remarkable advantages of rutin which include enhancement of solubility, protection from toxicity, bioavailability enhancement of pharmacological activity, and stability. These criteria have improved tissue macrophages distribution and protection from physical and chemical degradation. Also, reduce medicinal doses and improve the absorbency of herbal medicines compared with single therapy [83–86].

Clinical studies have supported effects as a cardioprotective and neuroprotective agent. The combination of polyphenols with existing drugs also shows promising results and significantly reduces their toxicity. The major limitation to the use of these plants is the side effects associated with their use in high doses due to their neurotoxic side effect and cardiac function, apoptosis, and necroptosis. During the clinical study, we reported a mixture of rutin, diosmin, troxerutin, hesperidin, and quercetin in the treatment of I–III degree hemorrhoidal disease in different time can effectively mean managing bleeding from hemorrhoidal disease and minimal adverse events [84, 87, 88].

## 4. Conclusion

This review summarizes that rutin can be a promising candidate in combination with drugs for cancer treatment *in vitro*. It has been shown that the antitumor effect of rutin is related to interactions with signalling processes such as mixed-lineage protein kinase 3, Wnt, and mitogen-activated protein kinase. Furthermore, it demonstrated that it inhibits cell proliferation and regulates apoptosis and cell cycle in cancer cell lines and helps to design the best therapeutic strategies. However, more future studies are needed to understand the proper mechanism of action of rutin on cancer cell lines. Also, further investigations are needed to assess rutin in combination or alone on the expression of anti- or proapoptotic pathways and genes and other ingredients.

## Figures and Tables

**Figure 1:** The structure of rutin and related flavonoids.

**Figure 2:** Regulation of activation of c-Fos and c-Jun proto-oncogenes on cancer cells.

**Figure 3:** Chemical structure of rutin (84).

**Figure 4:** Rutin can reduce the expression of proinflammatory cytokines (TNF-*α*, IL-6, IL-1*β,* and COX-2) and downregulate inflammatory markers and antiproliferative impact. This anti-inflammatory activity is primarily related to the regulation on MAPKs and NF-*κ*B signalling pathways by *in vivo* and *in vitro* data (66).

**Figure 5:** In a pathway independent of transcription, the mitochondrial *p*53 is bonded to Bcl-2 oncoprotein and Bcl-x proteins which reduce their inhibitory effect on the Bak and Bax apoptotic proteins. Bcl-2 promoted cell survival by blocking chemotherapy-induced apoptosis. Therefore, *p*53 leads to mitochondrial permeability and cytochrome C release consequently and activation apoptosis (21).

**Table 1:** The anticancer activities of rutin combination with other antioxidants or herbal ingredients.

Compound (rutin with other agents)	Mechanism	Cancer cell line	Reference
Quercetin, myricetin	Protection of cancer cells against hydrogen peroxide	Caco-2 and HepG2	[35, 36]
Quercetin	Decrease the activity of oxygen radical	Human hepatocellular carcinoma (HepG2)	[37–39]
AgNPs and natural bioactive compounds	Represent novel therapeutics fighting and synergistic, antimicrobial effects	Epithelioma papulosum cyprini (EPC) cell lines	[40]
Dietary polyphenols	Inducing cell cycle arrest or apoptosis, metastasis, and angiogenesis	Colorectal cancer cell lines	[41]
Fucoidan	Nuclear fragmentation, and mitochondrial potential loss, ROS generation	HaCaT (immortal noncancerous keratinocyte), HeLa (epithelial adenocarcinoma cells of the cervix)	[27]
Liquid crystalline nanoparticles	Inhibited the genes, namely, *Nox2B* and *Nox4*, which caused oxidative stress, upregulation in the expression of the antioxidant genes *Gclc* and *Nqo-1*	Human bronchial epithelial cells (BEAS-2B)	[36, 42]
Quercetin	Reduce the enzymes precarcinogenic compounds such as CYP1A	Intestinal HCT‐8 Cells	[38, 42]
Diosmin and Tangeretin	Antimetastatic effects	Melanoma B16F10 cancer cells	[43]
Zinc(II) flavonoid-metal complex	Modulated expression of genes related to angiogenesis, cell cycle progression	Leukaemia (KG1, K562, and Jurkat), melanoma (B16F10 and SK-Mel-28), and multiple myeloma (RPMI8226) cell lines	[44]
Ionic liquids nanoparticles	Caused a significant increase in the sub-G1 population, a significant decrease in cell viability	Human renal cancer cell line (786-O)	[45]
Silibinin	Anticancer, apoptosis effects regulating the expressions of genes apoptosis, inflammation, and MAPK pathway proteins	Human colon cancer cell line	[46]
Poly (D, L-lactic-co-glycolic acid) (PLGA) nanospheres, Benzamide	Cell cycle disruption and apoptotic induction	MDA-MB-231	[47]

**Table 2:** The anticancer activities of rutin combination with other therapeutically drugs as revealed by recent studies in vitro.

Compound (rutin with other therapeutically drugs)	Mechanism	Cancer cell line	Reference
Apigenin, tamoxifen	Induce apoptosis through a p53-dependent pathway	Breast cancer cell line (MCF-7)	[48]
Cisplatin, isoquercetin	Inducing toxicity, could decrees cell count percentage in G0/G1, S, and G2/M phases in addition to increase it in sub G0 phase in comparison with the single doses	Gastric cancer	[49]
Hyperoside	Increase the expression of regulator positive apoptosis such as Bax, Caspase 3, 8, 9	Colon cancer cells (HT-29)	[50]
5-FU	Increase of p53 gene expression and decreases Bcl-2 protein expression	Prostate cancer cell (PC3)	[21]
Oxaliplatin	Induced apoptosis may be associated with the activation of the p38/caspase signal pathway	SGC-7901 gastric cancer cell line	[51]
Orlistat	Cytotoxic effects and promoting apoptosis	Breast cancer (MCF-7) and pancreatic cancer cell line (PANC-1)	[5]
Oxidovanadium(IV)	Inhibit superoxide, hydroxyl radicals and improved the antioxidant activity	Lung cancer A549 cell line	[52]
5-FU and oxaliplatin	Antiproliferative effect and reduce possible adverse effects of these drugs	Caco-2 cancer cell line	[53]
Zein-*co*-acrylic acid hybrid hydrogels loaded 5-fluorouracil	Enhanced anticancer efficacy	MDA-MB-231 and MCF-7 breast cancer cell lines	[54, 55]
Doxorubicin (DOX)	Anticancer, protective effects	Human neuroblastoma cell line (IMR32)	[56]

## Data Availability

The data used to support the findings of this study are available from the corresponding author upon request.
